The article "Drug Flux Across RPE Cell Models: The Hunt for An Appropriate Outer Blood–Retinal Barrier Model for Use in Early Drug Discovery" was retracted in 2022. Reasons: contaminated cell lines or tissues; errors in the data; errors in the results or conclusions.

# Drug Flux Across RPE Cell Models: The Hunt for An Appropriate Outer Blood–Retinal Barrier Model for Use in Early Drug Discovery

**DOI:** 10.3390/pharmaceutics12020176

**Published:** 2020-02-19

**Authors:** Laura Hellinen, Heidi Hongisto, Eva Ramsay, Kai Kaarniranta, Kati-Sisko Vellonen, Heli Skottman, Marika Ruponen

**Affiliations:** 1 School of Pharmacy, Faculty of Health Sciences, University of Eastern Finland, 70210 Kuopio, Finland; laura.pelkonen@uef.fi (L.H.); kati-sisko.vellonen@uef.fi (K.-S.V.); 2 Department of Ophthalmology, Institute of Clinical Medicine, University of Eastern Finland, 70210 Kuopio, Finland; heidi.m.hongisto@tuni.fi (H.H.); kai.kaarniranta@uef.fi (K.K.); 3 Drug Research Programme, Division of Pharmaceutical Biosciences, Faculty of Pharmacy, University of Helsinki, P.O. Box 56, FI-00014 Helsinki, Finland; eva.ramsay@helsinki.fi; 4 Department of Ophthalmology, Kuopio University Hospital, P.O.Box 100, FI- 70029 Kuopio, Finland; 5 Faculty of Medicine and Health Technology, BioMediTech, Tampere University, 33520 Tampere, Finland; heli.skottman@tuni.fi

**Keywords:** retinal pigment epithelium, outer blood–retinal barrier, cell models, drug permeation, differentiation, tight junctions, ocular drug delivery

## Abstract

The retinal pigment epithelial (RPE) cell monolayer forms the outer blood–retinal barrier and has a crucial role in ocular pharmacokinetics. Although several RPE cell models are available, there have been no systematic comparisons of their barrier properties with respect to drug permeability. We compared the barrier properties of several RPE secondary cell lines (ARPE19, ARPE19mel, and LEPI) and both primary (hfRPE) and stem-cell derived RPE (hESC-RPE) cells by investigating the permeability of nine drugs (aztreonam, ciprofloxacin, dexamethasone, fluconazole, ganciclovir, ketorolac, methotrexate, voriconazole, and quinidine) across cell monolayers. ARPE19, ARPE19mel, and hfRPE cells displayed a narrow P_app_ value range, with relatively high permeation rates (5.2–26 × 10^−6^ cm/s. In contrast, hESC-RPE and LEPI cells efficiently restricted the drug flux, and displayed even lower P_app_ values than those reported for bovine RPE-choroid, with the range of 0.4–32 cm^−6^/s (hESC-RPE cells) and 0.4–29 × 10^−6^ cm/s, (LEPI cells). Therefore, ARPE19, ARPE19mel, and hfRPE cells failed to form a tight barrier, whereas hESC-RPE and LEPI cells restricted the drug flux to a similar extent as bovine RPE-choroid. Therefore, LEPI and hESC-RPE cells are valuable tools in ocular drug discovery.

## 1. Introduction

The retinal pigment epithelium (RPE) located in the posterior eye between the neural retina and choroidal circulation is essential for vision [1]. The RPE cell monolayer maintains the health of photoreceptors by regulating nutrient transport to and removing metabolic waste products from the subretinal space. Each day, the RPE cells also phagocytose shed photoreceptor outer segments, an important part of photoreceptor renewal. The RPE forms the outer blood-retinal barrier by forming tight junctions between the cells. This restricting barrier prevents the entry of xenobiotics into the eye, but also clinically useful drugs from the systemic blood circulation. In terms of intravitreal drug administration, RPE permeation is the main elimination route for small molecular-weight drugs [2]; however, it efficiently restricts macromolecular elimination, which means that these compounds have a longer elimination half-life in the vitreous [2,3]. The passage of drugs from the systemic circulation is restricted by the RPE, and thus only compounds with a high potency and/or selective targeting or a very wide therapeutic window can be administered systemically to treat retinal disorders. Ocular diseases, especially age-related macular degeneration, are becoming more common as the population ages [4]. These diseases represent a major burden for healthcare systems and discomfort for the patients. Ocular drug development against these retinal diseases is an area in which there is extensive research, but these programs demand reliable animal, tissue, and cell models, in order to improve the clinical relevance of early drug development.

The article "Drug Flux Across RPE Cell Models: The Hunt for An Appropriate Outer Blood–Retinal Barrier Model for Use in Early Drug Discovery" was retracted in 2022. Reasons: contaminated cell lines or tissues; errors in the data; errors in the results or conclusions.

Permeation across the RPE cell layer needs to be investigated when the ocular pharmacokinetics of new chemical entities is evaluated. The rabbit has been the most commonly used species in ocular pharmacokinetic studies [5,6]; however, simpler models, such as cells or isolated tissue sheets, are needed in early drug discovery when large numbers of molecules are screened. Currently, ex vivo models consisting of isolated RPE-choroid tissue sheets mounted in Ussing chambers are considered the most reliable outer blood–retinal barrier models in drug permeation studies [7]. The RPE-choroid tissue is usually isolated from the eyes of farm animals (porcine or bovine tissue) [2,8,9] as their tissue availability is better than that from humans. Due to the larger size of the eye, especially bovine eyes, the tissue extraction from these animals is easier than is the case in rabbits. However, tissue-sheet isolation from any species can be technically challenging and depending on the location of the abattoir or animal facility, the availability of freshly isolated eyes with a good tissue integrity can also be challenging.

RPE cells cultured on filter supports provide an alternative to isolated tissue sheets in permeation experiments. Several RPE cell models are available, with each having their own strengths and weaknesses. Human primary RPE cells are widely used in retinal biology studies, but they are rarely used in drug discovery. Due to the poor availability of adult human RPE cells, human fetal RPE cells (hfRPE) have been the most commonly used human primary RPE cell model. However, drug permeation across the primary RPE cells has not been reported.

The article "Drug Flux Across RPE Cell Models: The Hunt for An Appropriate Outer Blood–Retinal Barrier Model for Use in Early Drug Discovery" was retracted in 2022. Reasons: contaminated cell lines or tissues; errors in the data; errors in the results or conclusions.

The continuously growing human RPE cell line, ARPE19 [10], is the most widely used RPE model in the ocular drug discovery field, but it is leakier than bovine RPE-choroid [9,11]. The culture conditions and the phenotype of ARPE19 vary between laboratories, and the long differentiation required in specialized culture conditions is not ideal for high throughput screening. Another shortcoming of APRE19 cells is their lack of pigment - the native RPE is heavily pigmented and pigment binding is also a major factor in ocular pharmacokinetics, affecting both the drug distribution and retention in ocular tissues [12,13,14,15].

We have recently established two novel RPE cell models: ARPE19mel [16] and LEPI cells [17], which have advantageous properties in drug uptake and permeation experiments, respectively. ARPE19mel cells are artificially re-pigmented ARPE19 cells; the regular, non-pigmented ARPE19 cells are supplemented with functional melanosomes isolated from porcine RPE [18], leading to spontaneous phagocytosis and internalization of the pigmented organelles [16]. This cell model is valuable in studies focusing on the quantitative effects of pigmentation, such as drug uptake. LEPI cells, on the other hand, have spontaneously arisen from regular ARPE19 cultures. They have a distinct cobblestone morphology, rapid differentiation and doubling rates, and RPE-specific protein expression [17]. Importantly, we have previously demonstrated that this cell model reliably demonstrates the impact of permeant lipophilicity on membrane permeability and displays improved barrier properties by forming an even tighter barrier than the RPE-choroid [17].

In addition to clinical cell replacement therapy applications [19], the RPE cells differentiated from human embryonic (hESC) or human-induced pluripotent stem cells (hiPSC) are valuable in retinal research as they display a mature RPE phenotype after differentiation [20,21,22,23,24]. However, there is rather limited knowledge regarding the compound permeation of small molecular-weight compounds across hESC-RPE cells [25,26], and therefore, the applicability of hESC-RPE in early drug development is still unclear. Even though this cell model is considered to have perhaps the most appropriate RPE characteristics in culture, it has rarely been used in retinal drug research as cell differentiation is demanding and time consuming.

The article "Drug Flux Across RPE Cell Models: The Hunt for An Appropriate Outer Blood–Retinal Barrier Model for Use in Early Drug Discovery" was retracted in 2022. Reasons: contaminated cell lines or tissues; errors in the data; errors in the results or conclusions.

In summary, several RPE cell models are widely used in different fields of retinal research, but their barrier properties focusing on drug permeation have not been systematically compared within the same laboratory. In this paper, we present the permeation characteristics of nine small molecular-weight drugs with varying lipophilicities (logD_7.4_ values ranging from −5.1 to 1.92) across ARPE19, ARPE19mel, LEPI, hfRPE, and hESC-RPE cell monolayers. Importantly, in this study, we compared the obtained apparent permeation coefficients (P_app_) to the values recently obtained in our laboratory in an ex vivo bovine RPE-choroid model [2].

## 2. Materials and Methods

### 2.1. Cell Culture

**ARPE19 and LEPI cells.** ARPE19 cells (American Type Culture Collection, ATCC, Manassas, VA, USA, product CRL-2302) and LEPI cells [17] were maintained in our laboratory in DMEM/F-12 medium (Gibco, Thermo Fisher Scientific, Waltham, MA, USA) containing 10% fetal bovine serum (FBS, Gibco, Thermo Fisher Scientific, Waltham, MA, USA), 1% penicillin-streptomycin, and 2 mM L-glutamine (both products of Euroclone, Pero, Italy). The cells were seeded onto 1.12 cm^2^ polyester filters with a 0.4 µm pore size (3460-Clear Transwells, Corning Inc., Corning, NY, USA) at 160,000 cells/cm^2^, and cultured for 4 weeks in DMEM-F12 supplemented with 1% FBS, 1% penicillin-streptomycin, and 2 mM L-glutamine, before the experiments.

**ARPE19mel cells.** We have recently published a detailed description and characterization of re-pigmented ARPE19mel cells [16]. In the filter-culture format of ARPE19mel cells, the cells (ARPE19) were seeded onto filters as described above, and on the following day after seeding, functional melanosomes isolated from porcine RPE [18] were added to the growth medium, in the apical compartment. The pigment amount was quantified before the addition to achieve a melanosome amount equal to 1300 pg melanin/cell. This melanin content is similar to that present in intact porcine RPE [16]. The melanin amount was determined by an absorbance measurement (at 595 nm, Wallac Victor^2^ 1420 Multilabel counter, Perkin Elmer, MA, USA) utilizing isolated porcine RPE melanin standards (0.00–2.00 µg melanin/µL) [16,27]. Similar to the situation with regular ARPE19 cells, the ARPE19mel cells were cultured for 4 weeks before the experiments, in the same growth medium mentioned above.

**hfRPE cells.** The hfRPE cells were purchased from ScienCell (HRPEpiC cells, #6540 ScienCell, Carlsbad, CA, USA). The cells were expanded as reported previously [28], and seeded at a high density (200,000 cells/cm^2^) onto 1.12 cm^2^ Corning Transwell polyester inserts (3460-Clear Transwells, Corning Inc., Corning, NY, USA) at passage 3. The cells were cultured in EpiCM medium for 2 weeks before the permeation experiments (#4101, ScienCell, Carlsbad, CA, USA). We have previously provided a detailed characterization of these cells [28].

The article "Drug Flux Across RPE Cell Models: The Hunt for An Appropriate Outer Blood–Retinal Barrier Model for Use in Early Drug Discovery" was retracted in 2022. Reasons: contaminated cell lines or tissues; errors in the data; errors in the results or conclusions.

All the cells were cultured at +37 °C in 5% CO_2_, with the medium being replaced three times a week.

**hESC-RPE cells.** The hESC-RPE cells were differentiated from two genetically distinct hESC lines: Regea08/017 and Regea08/023. The derivation and characterization of the lines have been reported previously in [29]. Human ESCs were cultured on a Biolaminin 521 matrix (Biolamina, Sundbyberg, Sweden) in Essential 8 Flex Medium (Thermo Fisher Scientific, Waltham, MA, USA), as described in [23]. During RPE differentiation, hESCs were detached to make a single cell suspension with the TrypLE™ Select Enzyme (Tryple, Thermo Fisher Scientific, Waltham, MA, USA) and transferred to Corning^®^ Costar^®^ Ultra-Low attachment plates (Corning Inc., Corning, NY, USA) in RPEbasic medium containing KnockOut™ Dulbecco’s modified Eagle’s Medium supplemented with 15% KnockOut™ Serum Replacement, 2 mM GlutaMAX™, 1% MEM non-essential amino acids, 0.1 mM 2-mercaptoethanol, and 50 U/mL penicillin-streptomycin (all from Gibco, Thermo Fisher Scientific, Waltham, MA, USA). Embryoid body (EB) formation was induced by overnight induction with 10 μM blebbistatin (Sigma-Aldrich, St. Louis, MO, USA). For the following 2 days, EBs were allowed to undergo spontaneous differentiation in RPEbasic medium and on day 4, the EBs were plated down to 0.75 μg/cm^2^ LN-521 and 10 μg/cm^2^ human placental collagen type IV (col IV; Sigma-Aldrich, St. Louis, MO, USA) coating in RPEbasic medium. The medium was subsequently changed three times each week. After 30–45 days of differentiation, pigmented foci were selected with a scalpel, dissociated with Tryple, and re-plated in culture wells coated with LN-521 and col IV (RPE passage 1). Forty-five days later, the hESC-RPE was again re-plated (RPE passage 2) and then a further 9 days later, the hESC-RPE cells were frozen and subsequently thawed to final culture passage 3 in Corning^®^ Matrigel^®^ Matrix-coated (44 µg/cm^2^, cat. 356231, Corning Inc., Corning, NY, USA) PET inserts with a 1 µm pore size (cat. 83.3932.101 Sarstedt), with 250,000 cells/cm^2^. The hESC-RPE cells were cultured for 62 days prior to the permeation studies. The success of hESC-RPE cell differentiation was confirmed in detailed experiments; the RPE-specific properties of the differentiated cells are presented in Supplementary material in Figure S1 (characterization performed with the same procedures as described earlier in [23]).

The article "Drug Flux Across RPE Cell Models: The Hunt for An Appropriate Outer Blood–Retinal Barrier Model for Use in Early Drug Discovery" was retracted in 2022. Reasons: contaminated cell lines or tissues; errors in the data; errors in the results or conclusions.

Tampere University has the approval of the National Supervisory Authority for Welfare and Health (Valvira, Dnro 1426/32/300/05) to conduct research on human embryos. Tampere University also has supportive statements from the Ethical Committee of the Pirkanmaa Hospital District to derive, culture, and differentiate hESC lines (Skottman/R05116). No new hESC lines were derived in this study.

### 2.2. Permeation Studies

The permeation characteristics of aztreonam, ciprofloxacin, fluconazole, ganciclovir, ketorolac, methotrexate, quinidine, and voriconazole (Table 1) were evaluated as a cassette mix in both apical-to-basolateral (outward) and basolateral-to-apical (inward) directions. The drug concentration in the donor compartment was either 1 or 10 µg/mL (Table 1 in HBSS-Hepes (10 mM) buffer (pH 7.40)). The permeation was monitored for 3 h (ARPE19, ARPE19mel, hfRPE, and LEPI cells) or 6 h (hESC-RPE cells) at + 37 °C with low-speed shaking and the samples were collected at 15, 30, 45, 60, 75, 90, 120, 150, 180 (end-point for ARPE19, ARPE19mel, hfRPE, and LEPI cells), 210, 240, 270, 300, 330, and 360 min (end-point for hESC-RPE cells). The sample volumes were 0.5 mL in the basolateral and 0.2 mL in the apical compartment in the case of 1.12 cm^2^ filters and 0.35 mL in the basolateral and 0.1 mL in the apical compartment in the case of 0.3 cm^2^ filters.

The apparent permeation coefficient (P_app_ in cm/s) was determined with Equation (1) below:

P_app_ = J/(C_0_ × A), (1)

where J is the drug flux (ng/s) in the linear stage, C_0_ (ng/cm^3^) is the exposure concentration in the donor compartment, and A is the area (cm^2^) of the cell monolayer. The equation was valid if sink conditions were maintained, i.e., the receiver compartment concentration was below 10% of the concentration in the donor compartment.

The efflux ratios were calculated to determine the directionality of the drug permeation, using the following Equation (2):

Efflux ratio = P_app (apical-to-basolateral)_/P_app (basolateral-to-apical)._ (2)

### 2.3. Drug Concentration Measurements

The drug concentrations were determined with a liquid chromatograph (Agilent 1290, Agilent Technologies, Inc., Santa Clara, CA, USA) and a triple-quadrupole mass spectrometer (Agilent 6495; Agilent Technologies, Inc., Santa Clara, CA, USA) utilizing electrospray ionization in the positive ionization mode. We have previously described the method development and validation in detail [27,30], and a similar validation procedure was used in these LC-MS/MS runs.

The article "Drug Flux Across RPE Cell Models: The Hunt for An Appropriate Outer Blood–Retinal Barrier Model for Use in Early Drug Discovery" was retracted in 2022. Reasons: contaminated cell lines or tissues; errors in the data; errors in the results or conclusions.

## 3. Results

The P_app_ values, efflux ratios, and flux profiles are presented in detail in Supplementary material (Tables S1 and S2 and Figures S2 and S3).

We observed clear differences among the cell models in their barrier properties. A wide range of P_app_ values was observed in LEPI (0.4–29 *×* 10*^−^*^6^ cm/s) and hESC-RPE (0.4–32 *×* 10*^−^*^6^ cm/s) cells, similar to what was previously found in the bovine RPE-choroid that displayed P_app_ values for these drugs ranging from 1.4 to 69.2 *×* 10*^−^*^6^ cm/s (Figure 1A,B) [2]. There were up to 74-fold differences in these compounds’ P_app_ values in LEPI cells and 75-fold differences in hESC-RPE cells, demonstrating the intactness of the cell monolayers. In contrast, the P_app_ values of ARPE19, ARPE19mel, and hfRPE cells exhibited a very narrow range, only varying from 2.0 to 3.1-fold between compounds, and the values were all relatively high (5.2–26 *×* 10*^−^*^6^ cm/s, Figure 1A,B), reflecting the leakiness of the monolayers. In addition, the majority of the compounds permeated across ARPE19, ARPE19mel, and hfRPE in the apical-to-basolateral direction too rapidly to permit reliable P_app_ determination: the sink conditions were not maintained after the first hour (Supplementary material).

The lipophilic drug, fluconazole (logD_7.4_ 0.45), had P_app_ values in a similar range in all cells (varying between 5.4 and 25 *×* 10*^−^*^6^ cm/s, Figure 1C,D, Supplementary material), whereas the largest differences were seen with the hydrophilic compound, methotrexate (Figure 1E,F), with P_app_ values varying from 0.4 to 13 *×* 10*^−^*^6^ cm/s (Figure 1E,F, Supplementary material). Similarly, the P_app_ values of two other lipophilic compounds, quinidine (logD_7.4_ 1.17) and voriconazole (logD_7.4_ 1.21), were similar in all cell models (Figure 1A,B), whereas the more hydrophilic ganciclovir (logD_7.4_ −1.61) displayed 20-fold differences in its P_app_ values (range of 0.9–20 *×* 10*^−^*^6^ cm/s, Supplementary material).

Outward permeation values of methotrexate and ganciclovir were 4.4- and 2.9-fold higher, respectively, than inward permeation across the hESC-RPE cell line Regea08/017. Similarly, efflux ratios greater than 2 were observed for aztreonam (4.8), ciprofloxacin (3.9), ganciclovir (2.7), ketorolac (3.1), and methotrexate (3.0) across LEPI cells, i.e., evidence for a preference for the apical-to-basolateral (outward) direction (Table 2).

Compounds with a high affinity for melanin, i.e., ciprofloxacin and quinidine, displayed lag times of 100 and 200 min, respectively, in their permeation across hESC-RPE cells in the inward direction (Figure 2A,B). In the case of ciprofloxacin, the lag time of 100 min was similar to that present in the bovine RPE-choroid (Figure 2B). The flux profiles of ciprofloxacin and quinidine differed among ARPE19 and ARPE19mel cells (Figure 2C,D). These cells are otherwise identical, but ARPE19mel cells contain melanosomes [16].

The article "Drug Flux Across RPE Cell Models: The Hunt for An Appropriate Outer Blood–Retinal Barrier Model for Use in Early Drug Discovery" was retracted in 2022. Reasons: contaminated cell lines or tissues; errors in the data; errors in the results or conclusions.

## 4. Discussion

We performed a quantitative and systematic comparison of RPE cell model barrier functions by investigating drug flux across the cell monolayers of ARPE19, ARPE19mel, hfRPE, LEPI, and hESC-RPE cells. Our results clearly indicate that the hESC-RPE and LEPI cells restrict the drug permeation to a similar extent to that encountered in the ex vivo RPE model (bovine RPE-choroid), whereas ARPE19, ARPE19mel, and hfRPE cells display a leaky barrier, as indicated by the rapid drug flux and high P_app_ values. An overview of the cell model properties is presented in Table 3 below.

Permeation across the bovine RPE-choroid was recently investigated in our laboratory with eight small molecular-weight drugs: aztreonam, ciprofloxacin, fluconazole, methotrexate, ketorolac, quinidine, and voriconazole. The P_app_ values displayed a wide range: there was a 5-fold difference between the highly permeating lipophilic voriconazole and the slowly permeating hydrophilic aztreonam [2]. We observed a similarly wide range in the P_app_ values of hESC-RPE and LEPI cells, whereas the range of hfRPE, ARPE19, and ARPE19mel cells was narrow (Figure 1A,B). Because all the studied compounds displayed good permeation across the hfRPE, ARPE19, and ARPE19mel, these cells do not possess a tight barrier able to restrict drug permeation. The clearest differences between the leaky (hfRPE, ARPE19, and ARPE19mel) and tight (bRPE-choroid, hESC-RPE, and LEPI) epithelial barriers were seen with the hydrophilic compounds ganciclovir and methotrexate, which utilize the paracellular route (Figure 1A,B). Paracellular diffusion of these compounds is rapid across ARPE19, ARPE19mel, and hfRPE, indicating that their tight junctions are not able to efficiently restrict the drug flux.

The leakiness of the ARPE19 monolayer was an expected result: in the earlier work of Mannermaa et al. (2010), the cell line displayed a 7.6 times higher P_app_ value of hydrophilic 6-carboxyfluorescein, utilized as a paracellular marker, than bovine RPE-choroid [9,11]. However, ARPE19 cells reproduced the effect of a permeant size and lipophilicity on membrane permeation in that study, and therefore, the cell line can be a valuable tool in ocular drug research. In addition, ARPE19 cells display a similar transporter expression profile to primary RPE cells [28], suggesting that both of these cell models can be utilized in drug uptake studies. Furthermore, these leaky cell models might be suitable for predicting macromolecule or nanoparticle permeation across the RPE. It is possible that hfRPE and ARPE19 cells would develop a tighter barrier and a longer culture time in specialized culture conditions. ARPE19 cells can differentiate into a phenotype similar to adult RPE [31,32,33]; however, this can take several weeks or even months of differentiation. It should be noted that the addition of supplements (growth factors, sodium pyruvate, and amino acids) to ARPE19 growth media can lead to the creation of a tighter barrier due to multilayering of the cells instead of maturation of the tight junctions [11]. We observed the multilayering of hfRPE cells when an extracellular matrix (laminin or fibronectin) was used (data not shown), while culturing hfRPE cells on un-coated culture dishes resulted in a cell monolayer with an RPE-specific phenotype within 2 weeks [28,34]. In more advanced models, such as hESC-RPE, extracellular matrix coatings are routinely used. Human ESC-RPE cell differentiation, maturation, and barrier formation take several weeks in vitro and the extracellular matrix coating affects the barrier properties of the developing hESC-RPE cells [35]. Simple culture conditions were selected in this study for hfRPE cells and ARPE19-based models, since LEPI cells are able to differentiate rapidly, without the need for specialized culture conditions [17].

The article "Drug Flux Across RPE Cell Models: The Hunt for An Appropriate Outer Blood–Retinal Barrier Model for Use in Early Drug Discovery" was retracted in 2022. Reasons: contaminated cell lines or tissues; errors in the data; errors in the results or conclusions.

Stem-cell-derived RPE cells have been proven to differentiate into a phenotype that resembles adult RPE cells: the cells phagocytose photoreceptor outer segments; express various RPE-specific proteins; and display polarization, a high level of pigmentation, a polarized secretion of growth factors, and a tight barrier, as indicated by their tight junction protein expression and high transepithelial electrical resistance (TEER) [21,23,24]. The hESC-RPE cells were expected to form a tight barrier against drug diffusion as the permeation of 6-carboxyfluorescein was previously reported to be only slightly higher across hESC-RPE monolayers in comparison to bovine RPE-choroid (5–6-folds) [9,25]. This study confirmed that hESC-RPE cells display appropriate barrier characteristics against drug flux: the P_app_ values had a wide range and the cells restricted drug flux more efficiently than bovine RPE-choroid (Figure 1). The ARPE19-derived cell line LEPI restricted the drug flux to a similar extent as hESC-RPE cells, forming a tight epithelial barrier. We have previously characterized this cell line in detail; the cells display RPE-specific protein expression and functions [17].

The lipophilic compounds (fluconazole, voriconazole, and quinidine) displayed the highest permeation rates across bovine RPE-choroid, hESC-RPE, and LEPI cells, with similar P_app_ values in ARPE19 models and hfRPE cells (Figure S1, Supplementary material). This indicates that the permeation mechanism of fluconazole, quinidine, and voriconazole is transcellular passive permeation, as expected for lipophilic compounds. This finding highlights the importance of having appropriate model compounds when evaluating barrier formation: lipophilic compounds utilizing transcellular passive diffusion do not necessarily reveal the leakiness of the cellular barrier.

The article "Drug Flux Across RPE Cell Models: The Hunt for An Appropriate Outer Blood–Retinal Barrier Model for Use in Early Drug Discovery" was retracted in 2022. Reasons: contaminated cell lines or tissues; errors in the data; errors in the results or conclusions.

Directional permeation can be an indication of active transport, and efflux ratios outside the range of 0.5–2 point to the involvement of active transport [36]. We observed directionality in the permeation of methotrexate and ganciclovir in one of the hESC-derived RPE cell lines (Regea08/017) (Table 2); however, the efflux ratios were modest (4.4 and 2.9, respectively). In the case of LEPI cells, a directional preference in an outward direction was observed with hydrophilic compounds (aztreonam, ciprofloxacin, ganciclovir, ketorolac, and methotrexate, Table 2). These efflux ratios were also modest, ranging from 2.7 to 4.8. hESC-RPE and LEPI cells restricted the methotrexate and ganciclovir flux even more efficiently than bovine RPE-choroid (Figure 1E–F): P_app_ of methotrexate was 11.4-fold higher in the basolateral-to-apical direction across bovine RPE-choroid compared to hESC-RPE and LEPI, and the corresponding difference in ganciclovir P_app_ values was 6.6–7.4-fold, respectively. The poor permeation of ganciclovir and methotrexate can be explained by their physicochemical properties: hydrophilic compounds are not able to cross the cell monolayer transcellularly and tight junctions restrict the paracellular permeation. However, low permeation in both directions might partly be a consequence of active efflux on both sides of the RPE, and the minor directional differences can be caused by slight variations in the active transport rates. Ganciclovir is a substrate of MATE1 and methotrexate is a substrate of several transporter proteins, including MRP1, MRP4, and MRP5. Similarly, hydrophilic ketorolac is a substrate for OAT2 and both species differences between humans and cows and possible differences among the protein expression in human cell models can cause variation in the permeation, even between tight RPE models. All of the listed transporters have been detected at the protein level in RPE cell cultures [28,37]. A recent proteomics-based study indicated that these transporters are present on both RPE surfaces [34]. Passive permeation is expected to be the main permeation mechanism across the RPE for the majority of compounds, since an excellent correlation was observed between the physicochemical descriptors (hydrogen bonding and LogD_7.4_) and both intravitreal clearance [5] and systemic-to-eye drug transfer [38]. In addition, the impact of active transport in RPE permeation is expected to be low [39]. Our data supports this conclusion: most of the studied compounds did not display strong directional preferences, evidence of the predominance of passive permeation.

The article "Drug Flux Across RPE Cell Models: The Hunt for An Appropriate Outer Blood–Retinal Barrier Model for Use in Early Drug Discovery" was retracted in 2022. Reasons: contaminated cell lines or tissues; errors in the data; errors in the results or conclusions.

Differences in pigmentation are not expected to affect the compounds’ P_app_ values, but the linear phase in the drug flux across pigmented cells can be delayed in the case of melanin-bound compounds [9]. This is attributable to their larger intracellular volume of distribution. Ciprofloxacin and quinidine had dual-phased flux across highly pigmented hESC-RPE cells and bovine RPE-choroid (Figure 2A,B). Both ciprofloxacin and quinidine are high-melanin binders [27], and the lag times of 120–200 min needed to reach a steady-state in inward permeation can therefore be explained by melanin binding. The flux profile of quinidine did not show a clear lag time across the bovine RPE-choroid; however, the permeated amount was negligible (Figure 2A), and the mass balance was incomplete [2], which can be an indication of intracellular drug accumulation [2,9]. Since ARPE19-based cells had a leakier barrier, no clear lag time was observed with ARPE19mel cells. However, the flux profile of two high melanin-binders, i.e., ciprofloxacin and quinidine, is different in ARPE19 and ARPE19mel cells (Figure 2C,D), whereas the flux profiles of other drugs, all low melanin-binders [27], are similar in both cell lines (Supplementary material). Overall, non-pigmented cells can be utilized in permeation experiments as the P_app_ values are not dependent on the extent of pigmentation (Figure 1A,B). As pigment binding is a major factor affecting ocular pharmacokinetics [12,13], pigment binding properties need to be determined in early drug discovery; they can be determined with non-cellular binding studies [14,27,40] or with re-pigmented ARPE19mel cells [16].

Permeation across the RPE is an important parameter in ocular pharmacokinetics and thus needs to be screened during early drug development. In addition, realistic permeation values are crucial in in silico pharmacokinetic models. In this paper, we showed that hESC-RPE and LEPI cells display appropriate barrier properties against drug flux and are therefore valuable in vitro models in permeation experiments. Similar to Caco-2 cells and intestinal tissue [41], these RPE cells displayed even tighter barrier characteristics against drug flux than RPE-choroid tissue mounted in an Ussing chamber (Figure S1, Supplementary material). This finding is consistent with our earlier report in which we compared the permeation of beta-blockers across LEPI and bovine RPE-choroid [17]. LEPI cells are easily differentiated in simple culture conditions, making them a very attractive RPE cell model for high throughput screening, while advanced stem-cell-based models provide a platform on which to study permeation in disease-state cells [42].

The article "Drug Flux Across RPE Cell Models: The Hunt for An Appropriate Outer Blood–Retinal Barrier Model for Use in Early Drug Discovery" was retracted in 2022. Reasons: contaminated cell lines or tissues; errors in the data; errors in the results or conclusions.

## 5. Conclusions

In conclusion, our results reveal clear differences in the barrier function of RPE cell models. While useful in drug uptake studies, ARPE19-based models and hfRPE cells do not possess an appropriate barrier to restrict drug flux across the monolayer, whereas hESC-RPE and LEPI cells form a tight barrier comparable to bovine RPE-choroid. This difference was seen most clearly with hydrophilic compounds. The advantage of hESC-RPE cells is that they display lag-times with pigment-binding compounds due to the heavy pigmentation of these cells; however, their maintenance and differentiation are demanding and time-consuming. LEPI cells, on the other hand, are easily maintained and can be rapidly expanded and differentiated, making them an advantageous model for the outer blood–retinal barrier in assays requiring large numbers of cells, although they lack pigments. Overall, LEPI and hESC-RPE are clearly suitable outer blood–retinal barrier models for evaluating the permeation of small molecular-weight compounds.

## Figures and Tables

**Figure 1:** The studied retinal pigment epithelial (RPE) cell models display clear differences in their barrier properties. Both the outward (**A**) and inward (**B**) permeation of the drugs in ARPE19, ARPE19mel, and hfRPE cells lay in a narrow range, whereas in hESC-RPE and LEPI cells, there was a wide range of P_app_ values, similar to the situation in the bovine RPE-choroid (values from [2]). P_app_ values of the lipophilic drug fluconazole were similar among all the studied RPE models, indicating transport via a passive transcellular permeation route (**C**,**D**). The largest differences were observed in the permeation of the hydrophilic compound methotrexate (**E**,**F**), which displayed high permeation across ARPE19, ARPE19mel, and hfRPE cells, whereas in hESC-RPE cells, LEPI cells, and bovine RPE-choroid, its permeation was restricted more efficiently. n = 2–9, see Supplementary material for details. Abbreviations: n.a., not applicable (drug flux was too rapid for reliable P_app_ value determination: more than 10% of the compound permeated within 60 min).

The article "Drug Flux Across RPE Cell Models: The Hunt for An Appropriate Outer Blood–Retinal Barrier Model for Use in Early Drug Discovery" was retracted in 2022. Reasons: contaminated cell lines or tissues; errors in the data; errors in the results or conclusions.

**Figure 2:** Two high melanin-binders, quinidine and ciprofloxacin, display melanosomal accumulation in pigmented hESC-RPE and ARPE19mel cells. (**A**) Quinidine had a lag time of approximately 200 min in its permeation across the hESC-RPE cell layers, but no clear lag time was evident in bovine RPE-choroid (inset). (**B**) A permeation lag-time of approximately 100 min was detected for ciprofloxacin in hESC-RPE cells, which was similar to that present in bovine RPE-choroid (inset). Flux profiles of (**C**) quinidine and (**D**) ciprofloxacin differed between the non-pigmented ARPE19 and re-pigmented ARPE19mel cells. Number of replicates: ARPE19 and ARPE19mel, n = 3; hESC-RPE cells, n = 5; bovine RPE-choroid, n = 5 (quinidine) and n = 8 (ciprofloxacin).

**Table 1:** Compound information.

Compound	^1^ LogD_7.4_ (Predicted, ACDLabs)	Molecular Weight (g/mol)	^2^ Manufacturer	Exposure Concentration (µg/mL)
Aztreonam	−4.32	435.4	Fluka	10
Ciprofloxacin	−0.29	331.3	BioChemica	1
Dexamethasone	1.92	392.5	Sigma-Aldrich	10
Fluconazole	0.45	306.3	Sigma-Aldrich	1
Ganciclovir	−1.61	255.2	Sigma-Aldrich	1
Ketorolac	−0.34	255.3	Sigma-Aldrich	1
Methotrexate	-5.1	454.4	Fluka	1
Quinidine	1.17	324.4	Sigma-Aldrich	10
Voriconazole	1.21	349.3	Fluka	10

^1^ Values collected from the ChemSpider database (Royal Society of Chemistry) or from [2]. ^2^ Manufacturer locations: Fluka, USA; Biochemica, China; Sigma Aldrich, St. Louis, MO, USA.

**Table 2:** Efflux ratios of the studied compounds in tight RPE barriers.

Compound	LEPI	hESC-RPE (Regea08/017)	hESC-RPE (Regea08/023)	Bovine RPE-Choroid ^1^
Aztreonam	4.8	n.a.	n.a.	1.2
Ciprofloxacin	3.9	1.9	1.1	6.7
Dexamethasone	1.1	n.a.	n.a.	n.d.
Fluconazole	1.5	1.1	1.1	1.2
Ganciclovir	2.7	2.9	1.3	1.5
Ketorolac	3.1	1.8	1.3	14.5
Methotrexate	3.0	4.4	1.8	2.1
Quinidine	n.a.	0.9	0.7	n.a.
Voriconazole	n.a.	1.1	1.0	1.2

^1^ Values collected from [2]. n.a., P_app_ value could not be calculated due problems in analytics (aztreonam) or rapid drug flux (dexamethasone, quinidine, and voriconazole). n.d., not determined.

**Table 3:** Overview of the RPE cell model properties.

Cell Model	Culture Conditions	Tight Junction Protein Expression	Pigmentation	Barrier Properties: Conclusions of this Study	Assays in Which the Cell Model can be Utilized in Early Drug Discovery
**Cell lines**					
ARPE19	simple to demanding; variation between laboratories	yes	no	leaky	Drug uptake, active transport
ARPE19mel	simple	yes	can be controlled; from low to heavy	leaky	Drug uptake: quantitative effects of pigmentation
LEPI	simple	yes	no	tight	Drug uptake and permeation
**Primary RPE cells**					
hfRPE	simple	yes	low/modest	leaky	Drug uptake, active transport
**Stem-cell based RPE cells**					
hESC-RPE	demanding; long differentiation time, requires specialized conditions and expensive supplements	yes	heavy	tight	Drug uptake and permeation

The article "Drug Flux Across RPE Cell Models: The Hunt for An Appropriate Outer Blood–Retinal Barrier Model for Use in Early Drug Discovery" was retracted in 2022. Reasons: contaminated cell lines or tissues; errors in the data; errors in the results or conclusions.

## Supplementary Materials

The following are available online at https://www.mdpi.com/1999-4923/12/2/176/s1: Supplementary Materials: The characterization of hESC-RPE cultures and P_app_ values, efflux ratios, and flux profiles for each cell model and studied compound (PDF-file). Figure S1: Human ESC-RPE cells display characteristic RPE properties prior to the permeation studies; Figure S2: Flux of hydrophilic compounds across RPE cell models and bovine RPE-choroid; Figure S3: Flux of lipophilic compounds across RPE cell models and bovine RPE-choroid; Table S1: Apparent permeation coefficients; Table S2: Efflux ratios.
